# Discrete Two-Step Cross-Modal Hashing through the Exploitation of Pairwise Relations

**DOI:** 10.1155/2021/4846043

**Published:** 2021-09-27

**Authors:** Shaohua Wang, Xiao Kang, Fasheng Liu, Xiushan Nie, Xingbo Liu

**Affiliations:** ^1^College of Electrical Engineering and Automation, Shandong University of Science and Technology, Qingdao, China; ^2^School of Software, Shandong University, Jinan, China; ^3^School of Computer Science and Technology, Shandong Jianzhu University, Jinan, China

## Abstract

The cross-modal hashing method can map heterogeneous multimodal data into a compact binary code that preserves semantic similarity, which can significantly enhance the convenience of cross-modal retrieval. However, the currently available supervised cross-modal hashing methods generally only factorize the label matrix and do not fully exploit the supervised information. Furthermore, these methods often only use one-directional mapping, which results in an unstable hash learning process. To address these problems, we propose a new supervised cross-modal hash learning method called Discrete Two-step Cross-modal Hashing (DTCH) through the exploitation of pairwise relations. Specifically, this method fully exploits the pairwise similarity relations contained in the supervision information: for the label matrix, the hash learning process is stabilized by combining matrix factorization and label regression; for the pairwise similarity matrix, a semirelaxed and semidiscrete strategy is adopted to potentially reduce the cumulative quantization errors while improving the retrieval efficiency and accuracy. The approach further combines an exploration of fine-grained features in the objective function with a novel out-of-sample extension strategy to enable the implicit preservation of consistency between the different modal distributions of samples and the pairwise similarity relations. The superiority of our method was verified through extensive experiments using two widely used datasets.

## 1. Introduction

With the development of Internet technology in recent years, a large quantity of multimodal data obtained from video, audio, image, text, and other sources are being disseminated rapidly across social networks. A common requirement in real scenarios is cross-modal retrieval, e.g., retrieving corresponding images or videos through text descriptions. Owing to the heterogeneity of multimodal data, cross-modal retrieval tasks must, unlike traditional retrieval tasks, bridge the semantic gap and acquire common and unified expressions. At the same time, the rapidly growing mass of data has increased the time and space costs of retrieval to serve users who generally expect to be able to quickly obtain information related to their retrieval targets.

Owing to its high retrieval efficiency and low space cost, cross-modal hashing has become one of the primary methods in the field of cross-modal retrieval [1]. Cross-modal hash learning attempts to convert multimodal data into a set of short binary codes (called hash codes) in Hamming space while preserving the original sample relations and then to learn a set of mapping functions from the specific modality to the sample hash code. The binary code of the common space and the mapping from the specific modality to the common space can be used to achieve cross-modal retrieval. As the similarities between hash codes are calculated as Hamming distances, the XOR operation can be implemented on hardware to significantly improve retrieval efficiency. Furthermore, the storage cost is reduced because the hash code length is relatively short.

The existing cross-modal hashing approaches can be roughly divided into unsupervised and supervised methods. Unsupervised methods learn hash functions by exploiting the sample relations between and within modalities, which often have low accuracies. Supervised methods attempt to exploit the supervision information contained in labels and use the common semantic information in these labels to guide the learning of the hash code, thereby improving its quality. However, most existing supervised methods do not fully exploit the supervision information [2, 3]. For example, Xu et al. [4] used label matrix regression alone and ignored the similarity relations between samples. Furthermore, the one-directional regression used by supervised methods is not conducive to the full exploitation of supervision information and will also cause the hash learning process to be unstable. Therefore, in this paper we propose a new supervised cross-modal hashing method that combines label matrix factorization and hash code regression to achieve bidirectional mapping. In addition, a dual supervision approach is adopted to embed the label and pairwise similarity matrices into the hash learning process to further exploit the pairwise relations between modalities.

Another important problem in hash learning is the integer optimization problem caused by binary constraints. The introduction of the pairwise similarity matrix has made the optimization of the objective function more complicated. Currently available methods generally adopt a relaxation strategy in which the binary constraint is abandoned; instead, the real value is optimized and the thresholding method is then used to obtain a solution. However, this method will cause cumulative quantization errors. In this work, we propose a semirelaxed, semidiscrete strategy to minimize quantization errors and improve retrieval accuracy while ensuring the smooth optimization of the objective function. Furthermore, inspired by the concept of heterogeneous modal feature fusion under the bilinear model [5], we propose a simple mapping learning to fuse multimodal data to obtain more fine-grained high-order features, which are used in combination with the proposed out-of-sample extension strategy to implicitly preserve the similarity relations between samples.

In summary, the contributions of this study are as follows:

- A new cross-modal supervised hashing framework using dual supervision information is designed to exploit the pairwise relations between samples. Furthermore, a semirelaxed and semidiscrete strategy is adopted to exploit the pairwise similarity matrix to reduce cumulative quantization errors.
- A new out-of-sample extension strategy with two novel optimization strategies is developed. By combining this strategy with the fine-grained features, the consistency between the different sample modal distributions and the pairwise similarity relations can be effectively preserved.
- Experiments were conducted on two widely used retrieval datasets to verify the effectiveness and superiority of the proposed method.

The remainder of the article is organized as follows.  Section 2 briefly reviews some related works.  Section 3 gives the details of DTCH.  Section 4 presents the experimental results and discussions, followed by the conclusion in Section 5.

## 2. Related Work

The currently available cross-modal hashing methods can be primarily divided into linear model-based [6–8] and deep model-based [9–12] methods. Although some recently proposed methods based on deep models have improved retrieval performance, such approaches generally exhibit high time and space complexities and have poor interpretabilities. By contrast, linear models are more applicable to real scenarios owing to their high retrieval efficiencies and strong interpretabilities.

The existing linear cross-modal retrieval methods can be further divided into two main categories: unsupervised cross-modal hashing [13–15] and supervised cross-modal hashing [16–19]. The unsupervised cross-modal hashing methods primarily learn hash functions by mining sample feature information to obtain relations between and within sample modalities. For example, Sun et al. [13] extended the traditional spectral hashing approach to the multimodal field by minimizing the Hamming distances between sample pairs. Intermedia hashing [14] learns hash codes by maintaining the semantic consistencies between and within modalities. Zhou et al. [15] proposed a latent semantic sparse hashing method in which matrix factorization and sparse coding are combined to discover a common Hamming space.

In contrast to the unsupervised learning methods, the supervised cross-modal hashing methods use label information and pairwise similarity information to improve hash code quality. Zhang et al. [16] used the pairwise similarity matrices generated from labels to learn hash codes and then attempted to use these hash codes to reconstruct the matrices with the goal of maximizing the semantic correlations of the hash codes. Xu et al. [4] extended supervised discrete hashing (SDH) [20] to the cross-modal field and used the label matrix regression method to directly learn hash codes. However, SDH adopts the bitwise learning strategy to generate binary codes, making it time-consuming. Chen et al. [17] proposed a scalable cross-modal hashing method in which matrix factorization is applied to the cross-modal field. Generally speaking, the retrieval accuracies of supervised learning methods are significantly higher than those of unsupervised methods owing to the exploitation of label information. In general, these methods are restricted by their weak representation ability. To obtain satisfactory accuracy, longer code lengths are often required, leading to greater storage and query costs.

## 3. Proposed Method

In this section, we introduce our method in detail in terms of its use of notation, binary code learning, optimization, out-of-sample extension, and time complexity. The framework is shown in Figure 1.

### 3.1. Notation

For a dataset **X**={*v*_*i*_, *t*_*i*_}_*i*=1_^*N*^ with *N* sample pairs, we use *v*_*i*_ ∈ *R*^*d*^ to represent the eigen vector of the image modality in the i-th sample pair and *t*_*i*_ ∈ *R*^*d*^ to represent the eigen vector of the text modality in the *i*-th sample pair, where *d* and *f* are the corresponding eigen dimensions. Correspondingly, **V** ∈ *R*^*d*×*N*^ and **T** ∈ *R*^*f*×*N*^ represent the visual modal feature and the text modal matrices, respectively. In addition, **Y** is used to represent the sample label matrix, where **y**_*i*_={*y*_*ic*_} ∈ {0,1}^*C*^ represents the label vector corresponding to the *i*_th_ sample, where *C* represents the number of classes. If the current sample **x**_*i*_ belongs to the *c*_th_ class, then *y*_*ic*_=1, where *c*=1,…, *C*; otherwise, *y*_*ic*_=0. At the same time, the label matrix **Y** is used to construct the pairwise similarity matrix **S** ∈ {−1, +1}^*N*×*N*^. If the sample pair *i* and *j* are similar, then *S*_*i*,*j*_=1; otherwise, *S*_*i*,*j*_=−1.

### 3.2. Binary Code Learning

The goal of cross-modal hashing is to map heterogeneous multimodal data onto compact binary codes while preserving the semantic similarity of the original space. Intuitively, multimodal data describe the same entity and, therefore, their high-level semantics should be consistent. This paper proposes a new cross-modal hashing framework that fully exploits the pairwise relations of samples contained in the label and pairwise similarity matrices to learn a unified binary code.

Inspired by Multimodal Discriminative Binary Embedding (MDBE) [21], we attempted to use matrix factorization to explore the semantic information implicit in the label matrix. This process can be formalized as follows:

(1) $$\begin{array}{c} \underset{M,B}{\min}{\left\|Y-BM\right\|}^{2}+\lambda {\left\|M\right\|}^{2}\\ \text{s.t.}\;B\in {\left\{-1,1\right\}}^{N\times L}, \end{array}$$

where **B** ∈ {−1,1}^*N*×*L*^ is the binary semantic representation learned from the label matrix, i.e., the hash code, and *M* is the auxiliary matrix. To avoid singular solutions, we add the *L*_2_-norm regularization term to **M**. In addition, by regressing the label matrix to the hash code, the label matrix can be embedded into the learning of the binary code as follows:

(2) $$\begin{array}{c} \underset{W,B}{\min}{\left\|B-YW^{T}\right\|}^{2}+\lambda {\left\|W\right\|}^{2}\\ \text{s.t.}\;B\in {\left\{-1,1\right\}}^{N\times L}, \end{array}$$

where **W** is the linear mapping matrix. In addition to further exploration of the semantic information in the label matrix, equation (2) can be used to stabilize the hash learning process. The full exploitation of the label matrix can reduce the semantic gap caused by modal heterogeneity to the greatest extent possible, making it more likely that the hash code expresses high-level semantics beyond the specific modal. In other words, the label information is not restricted by the specific modality and the hash code learned from label information should be a more advanced representation that can cross the semantic gap.

Additional important supervision information for the supervised hash learning method is obtained from the pairwise similarity matrix. A common approach to constructing the pairwise similarity matrix for the cross-modal supervised hashing method is to reconstruct the sample label matrix. If two sample pairs share one or more labels, they are considered similar, and vice versa. As the inner product of the hash code between two samples corresponds to the distance between the samples, it can be used as a measure of the similarity relation between the samples. Therefore, the inner product of the hash code is used to fit the pairwise similarity matrix to ensure that the learned hash code maintains the similarity relations of the original space as much as possible, which is consistent with the original intention of cross-modal hash learning. This process can be modeled as follows:

(3) $$\begin{array}{c} \underset{B}{\min}{\left\|BB^{T}-L\cdot S\right\|}^{2}\\ \text{s.t.}\;B\in {\left\{-1,+1\right\}}^{N\times L}, \end{array}$$

where **B** ∈ {−1,1}^*N*×*L*^ is the binary semantic representation learned from the label matrix, i.e., the hash code, and *L* denotes the length of hash code. Clearly, equation (3) is a nonconvex optimization problem that is difficult to solve. Many existing methods have adopted a complete relaxation strategy involving the removal of the discrete constraint on the hash code. However, this approach will produce accumulated quantization errors that seriously affect the accuracy of hash retrieval. To solve this problem, we adopt a semidiscrete, semirelaxed strategy in which the real value information in equation (2) is used to replace the hash matrix *B* in equation (3). In this manner, the rich semantic information in the real value can be fully exploited without destroying the discrete constraints on the hash code. This process can be formalized as follows:

(4) $$\begin{array}{c} \underset{B,W}{\min}{\left\|BWY^{T}-S\right\|}^{2}\\ \text{s.t.}\;B\in {\left\{-1,+1\right\}}^{N\times L}. \end{array}$$

According to the bilinear model [5], high-order features obtained through the fusion of heterogeneous features can better characterize an original sample. Inspired by this idea, the proposed approach fuses data obtained from different modalities. It is worth noting that because different modal data exist in different feature spaces, there will be semantic gaps between them. Therefore, a simple feature mapping must be learned prior to fusion to aid in the feature space transformation, that is, **VPT**^*T*^. Further, by combining this formulation with equation (4), this fine-grained feature can be embedded into hash learning as follows:

(5) $$\begin{array}{c} \underset{B,W,P}{\min}{\left\|BWY^{T}-V^{T}PT\right\|}^{2}\\ \text{s.t.}\;B\in {\left\{-1,+1\right\}}^{N\times L}, \end{array}$$

where **V** and **T** are features of different modalities and **P** is the linear projection. This equation reinforces the learning of hash codes using the fine-grained features **VPT**^*T*^ and improves the quality of the hash codes. At the same time, it can be applied in conjunction with the out-of-sample extension strategy to produce learned hash codes for different modal samples that preserve the pairwise similarity relations as much as possible, as will be introduced in detail in Section 3.4.

In summary, by combining equations (1), (2), (4), and (5), the final objective function can be obtained as follows:

(6) $$\begin{array}{c} \underset{M,W,B,P}{\min}{\left\|Y-BM\right\|}^{2}+\alpha {\left\|B-YW^{T}\right\|}^{2}+\beta {\left\|BWY^{T}-V^{T}PT\right\|}^{2}+\gamma {\left\|BWY^{T}-S\right\|}^{2}+\lambda \left({\left\|M\right\|}^{2}+{\left\|W\right\|}^{2}\right)\\ \text{s.t.}\;B\in {\left\{-1,1\right\}}^{N\times L}, \end{array}$$

where *α*, *β*, *γ*, and *λ* are tradeoff parameters.

### 3.3. Optimization

Equation (6) is evidently still a difficult-to-solve nonconvex optimization problem for variables **W**, **B**, **M**, and **P**. However, solving for a single variable while fixing the other variables remains a relatively straightforward process. Therefore, we propose an alternating iteration strategy for optimization with the goal of achieving global optimization through local optimization. Each optimization step is introduced as follows:

  Step 1: first, the optimization process of the mapping **M** is introduced. By fixing the remaining three variables, equation (6) can be simplified to

(7) $$\begin{array}{c} \underset{M}{\min}{\left\|Y-BM\right\|}^{2}+\lambda {\left\|M\right\|}^{2}. \end{array}$$

  By taking the derivative of equation (7) with respect to **M** and setting it equal to zero, we obtain

(8) $$\begin{array}{c} B^{T}BM+\lambda M=B^{T}Y. \end{array}$$

  By solving the above equation, the closed-form (analytical) solution of **M** can be obtained as follows:

(9) $$\begin{array}{c} M={\left(B^{T}B+\lambda I\right)}^{-1}B^{T}Y. \end{array}$$

  Step 2: fix the three variables **M**, **B**, and **P**, and optimize the mapping **W**. In this case, the objective function can be simplified to

(10) $$\begin{array}{c} \underset{W}{\min}\alpha {\left\|B-YW^{T}\right\|}^{2}+\beta {\left\|BWY^{T}-V^{T}PT\right\|}^{2}+\gamma {\left\|BWY^{T}-S\right\|}^{2}+\lambda {\left\|W\right\|}^{2}. \end{array}$$

  By taking the derivative of equation (10) with respect to **W** and setting it equal to zero, we obtain

(11) $$\begin{array}{c} \alpha WY^{T}Y+\left(\beta +\gamma \right)B^{T}BWY^{T}Y=\alpha B^{T}Y+\beta B^{T}V^{T}PTY+\gamma B^{T}SY. \end{array}$$

  The closed-form solution of **W** is

(12) $$\begin{array}{c} W={\left(\alpha I+\left(\beta +\gamma \right)B^{T}B\right)}^{-1}\left(\alpha B^{T}Y+\beta B^{T}VPT^{T}Y+\gamma B^{T}SY\right){\left(Y^{T}Y\right)}^{-1}. \end{array}$$

  Step 3: optimize variable **B**. By fixing the remaining variables, we obtain

(13) $$\begin{array}{c} \underset{B}{\min}{\left\|Y-BM\right\|}^{2}+\alpha {\left\|B-YW^{T}\right\|}^{2}+\beta {\left\|BWY^{T}-V^{T}PT\right\|}^{2}+\gamma {\left\|BWY^{T}-S\right\|}^{2}\\ \text{s.t.}\;B\in {\left\{-1,1\right\}}^{N\times L}. \end{array}$$

  As **B** contains binary constraints, equation (13) is still an integer optimization problem. Here, we introduce two approaches to optimizing **B**. The first optimization scheme uses discrete proximal linearized minimization (DPLM) [22]. After reconstruction and simplification, **B** can be solved through a simple symbolic function:

(14) $$\begin{array}{c} B^{j+1}=\mathrm{sgn}\left(B^{j}-\frac{1}{\mu }▽L\left(B^{j}\right)\right), \end{array}$$

  where **B**^*j*^ is the solution of **B** after the *j*_th_ iteration, *μ* is a hyperparameter, and ▽*L*(**B**) is expressed as follows:

(15) $$\begin{array}{c} ▽L\left(B\right)=BMM^{T}+\left(\beta +\gamma \right)BWY^{T}YW^{T}-YM^{T}-\alpha YW^{T}-\beta VPT^{T}YW^{T}-\gamma SYW^{T}. \end{array}$$

  The second optimization scheme for **B** adopts the discrete cyclic coordinate descent (DCC) approach [20]. Although equation (13) is an integer optimization problem, the DCC algorithm can still be employed to solve its discrete solution iteratively and bit by bit. As ‖**B**‖^2^=*L∗N*, equation (13) can be rewritten as

(16) $$\begin{array}{c} \underset{B}{\min}{\left\|MB^{T}\right\|}^{2}+\left(\beta +\gamma \right){\left\|BWY^{T}\right\|}^{2}-\text{Tr}\left(B^{T}Q\right)\\ \text{s.t.}\;B\in {\left\{-1,+1\right\}}^{N\times L}, \end{array}$$

  where **Q**=**YM**^*T*^+*α ***YW**^*T*^+*β ***SYW**^*T*^+*γ ***VPT**^*T*^**YW**^*T*^. According to the DCC algorithm, we define **b** as the *l*-th column of matrix **B**, *l*=1,…, *L*, and *B*′ as matrix **B** excluding **b**. Analogously, we define **q** as the *l*-th column of matrix **Q**. We then define **m** as the *l*-th column of matrix **M** and *M*′ as matrix **M** excluding **m**. Finally, we define *H*=**WY**^*T*^, **h** as the *l*-th column of matrix **H**, and *H*′ as matrix **H** excluding **h**. Equation (16) can then be rewritten as

(17) $$\begin{array}{c} \underset{b}{\max}b^{T}\left(q-B^{\prime }M^{\prime }m-\left(\beta +\gamma \right)B^{\prime }H^{\prime }h\right)\\ \text{s.t.}\;b\in {\left\{-1,+1\right\}}^{N\times L}. \end{array}$$

  By taking the derivative, the analytical solution of **b** can be obtained as follows:

(18) $$\begin{array}{c} b=\text{sign}\left(q-B^{\prime }M^{\prime }m-\left(\beta +\gamma \right)B^{\prime }H^{\prime }h\right), \end{array}$$

  where sgn(·) represents the symbolic function.
  Step 4: fix the remaining variables and optimize mapping **P**. In this case, the objective function is

(19) $$\begin{array}{c} \underset{P}{\min}{\left\|BYW^{T}-V^{T}PT\right\|}^{2}. \end{array}$$

By taking the derivative and setting it equal to zero, we obtain

(20) $$\begin{array}{c} VV^{T}PTT^{T}-VBWY^{T}T=0. \end{array}$$

The closed-form solution of **P** is

(21) $$\begin{array}{c} P={\left(VV^{T}\right)}^{-1}VBWY^{T}T{\left(TT^{T}\right)}^{-1}. \end{array}$$

### 3.4. Out-of-Sample Extension

In this section, we introduce the out-of-sample extension strategy. As shown in equation (6), DTCH is a two-step hashing method. After the offline training is completed, a mapping from features to hash codes must also be learned to query the samples. As mentioned above, we propose a new out-of-sample extension strategy that, when combined with the objective function, can help ensure that the learned modality-specific out-of-sample mappings **P**_*V*_ and **P**_*T*_ preserve the similarity in the original space. Specifically, this strategy can be formalized as follows:

(22) $$\begin{array}{c} \underset{P_{V},P_{T}}{\min}{\left\|B-VP_{V}\right\|}^{2}+{\left\|B-TP_{T}\right\|}^{2}+\sigma {\left\|{\left(VP_{V}\right)}^{T}TP_{T}-S\right\|}^{2}, \end{array}$$

where the solution of the out-of-sample extension mapping for the visual modality can be expressed as

(23) $$\begin{array}{c} \underset{P_{V}}{\min}{\left\|B-VP_{V}\right\|}^{2}+\sigma {\left\|{\left(VP_{V}\right)}^{T}TP_{T}-S\right\|}^{2}. \end{array}$$

By taking the derivative with respect to **P**_*V*_, we obtain

(24) $$\begin{array}{c} P_{V}={\left(V^{T}V+\sigma V^{T}TP_{T}P_{T}^{T}T^{T}V\right)}^{-1}\left(V^{T}B+\sigma V^{T}STP_{T}\right). \end{array}$$

The solution of the out-of-sample extension mapping for the text modality can be expressed as

(25) $$\begin{array}{c} \underset{P_{T}}{\min}{\left\|B-TP_{T}\right\|}^{2}+\sigma {\left\|{\left(VP_{V}\right)}^{T}TP_{T}-S\right\|}^{2}. \end{array}$$

By taking the derivative with respect to **P**_*T*_, we obtain

(26) $$\begin{array}{c} P_{T}={\left(T^{T}T+\sigma T^{T}VP_{V}P_{V}^{T}V^{T}T\right)}^{-1}\left(T^{T}B+\sigma T^{T}SVP_{V}\right). \end{array}$$

### 3.5. Time Complexity

In the training process, we need to update the projection **M**, **W**, **P**, **P**_*V*_, and **P**_*T*_ and the unified binary code matrix **B**. The time complexity for learning **M**, **W**, and **P**, **P**_*V*_, and **P**_*T*_ are *O*(2*f*^2^*N*+2*d*^2^*N*+LdN+LfN), *O*(*N*^2^*L*+NL^2^+NC^2^), *O*(NdL+NfL+*f*^2^*N*+*d*^2^*N*), and *O*(*N*^2^*d*+*N*^2^*f*), respectively. In this study, we adopt two approaches to optimize **B**. Specifically, solving equations (15) and (18) requires *O*(NL^2^+LdN+LfN) and *O*(LdCN^2^+LfCN^2^), respectively. As *N* is usually much larger than *C* and *L*, the training time complexity of the proposed method with DCC and DPLM can be simplified as *T* · *O*(2*N*^2^*L*+*N*^2^*d*+*N*^2^*f*) and *T* · *O*(LdCN^2^+LfCN^2^+*N*^2^*L*+*N*^2^*f*), where *T* is the number of iterations.

## 4. Experiments

To verify the effectiveness of the proposed method, we conducted extensive experiments using two widely used datasets. In the following section, the three aspects of each dataset (their modalities and class information) experimental settings, and experimental analyses and results are introduced in detail.

### 4.1. Dataset

To verify the effectiveness and superiority of the proposed method, we conducted extensive experiments using two widely used large-scale cross-modal retrieval datasets: MIR-Flickr [23] and NUS-WIDE [24].

The MIR-Flickr dataset contains 25,000 images in 24 classes, with each image forming an image-text pair with a corresponding text description. In this study, 15,902 sample pairs were selected as the training set, 836 sample pairs were selected as the test set, and the union of these sets was used as the retrieval set. Specifically, the image modality was represented by a 150-dimensional edge histogram, the text modality was represented by a 500-dimensional word vector, and the class information was represented by a 24-dimensional semantic label.

The NUS-WIDE dataset contains 269,648 images and corresponding text descriptions from the Internet and includes 81 classes. In this study, the 10 most frequent classes and their 17,000 corresponding samples were selected for training, 994 samples were selected for testing, and 50,000 samples were selected for retrieval. Specifically, the image modality was represented by a 500-dimensional SIFT bag-of visual words vector [25], the text modality was represented by a 1,000-dimensional bag-of-words vector, and the class information was represented by a 10-dimensional semantic label.

### 4.2. Experimental Settings

Using the two datasets described above, we compared DTCH with eight cross-modal hashing methods that have been proposed in recent years: cross-view hashing (CVH) [13], intermedia hashing (IMH) [14], latent semantic sparse hashing (LSSH) [15], semantic correlation maximization (SCM) [16], discrete cross-modal hashing (DCH) [4], fast discrete cross-modal hashing (FDCH) [26], scalable discrete matrix factorization hashing (SCRATCH) [17], and two-step cross-modal hashing (TECH) [18]. Among these, CVH, IMH, and LSSH are unsupervised methods and the others are supervised methods.

For a fair comparison, the hyperparameters of all baseline methods were initialized according to the approaches used in the original papers; for all methods, including DTCH, the average performance over five runs was used for comparison. The following parameter settings were used for the method proposed in this paper: *α*=2, *β*=10^−7^, *γ*=10^−7^, *λ*=10^−4^, *μ*=0.05, and *σ*=10^−7^. As the proposed method is based on a linear model, a deep model was not used as its baseline method. Moreover, all examinations are led on a computer with an Intel Core i7-6700 3.40 GHz 4 processor and 32 GB RAM under the programming climate of MATLAB R2019b.

To compare the performance of the methods, we tested each on two cross-modal retrieval tasks: (1) Img2Text, involving the retrieval of texts using images; and (2) Text2Img, involving the retrieval of images using texts. The average precision (AP) and mean average precision (mAP) were used as metrics. AP represents the average precision of to-be-retrieved samples as follows:

(27) $$\begin{array}{c} \text{AP}=\frac{1}{D}\sum_{r=1}^{K}\text{Precision}\left(r\right)\sigma \left(r\right), \end{array}$$

where *D* is the number of correlated samples among K retrieved samples and *σ*(*r*) indicates whether the *r*_th_ example is correlated with a retrieved sample. mAP was obtained by sorting the AP values of the samples and then taking the average as follows:

(28) $$\begin{array}{c} \text{mAP}=\frac{1}{Z}\sum_{r=1}^{Z}\text{AP}\left(i\right), \end{array}$$

where *Z* represents the number of samples to be retrieved.

### 4.3. Experimental Results and Analyses

In this section, we provide a brief analysis of the experimental results.  Table 1 lists the mAP scores of the cross-modal retrieval results obtained by applying DTCH and the eight comparison methods to the two datasets, MIR-Flickr and NUS-WIDE. The upper half of the table lists the result performances obtained in applying Img2Text; the lower half lists the Text2Img result performances. Ours-1 and Ours-2 adopted DCC and DPLM, respectively, for solution optimization. It is seen from Table 1 that Ours-2 achieved the best performance under various code lengths on both datasets, indicating that the proposed method was able to reduce the semantic gap to a certain extent and improve the cross-modal retrieval performance. Ours-1 also obtained convincing results; in performing the Text2Img task in particular, its performance was significantly improved relative to the previous methods. On the NUS-WIDE dataset, however, the performance of Ours-1 was slightly worse than that of SCARTCH, particularly at relatively short code lengths. One possible reason for this result is that Ours-1 was trapped in local optima while using DCC optimization. In addition, its insufficient performance on the Img2Text task alone indicates that its characterization ability on the image modality is slightly lacking. Thus, in subsequent work it will be useful to enhance the image modal expression ability of the proposed method.

Figure 2 shows a line chart plotting the average Precision@K indicator as a function of code length for each method in performing each task. Without loss of generality, the value of *K* was selected to be 50. It is seen from the results that Ours-1 and Ours-2 achieved optimal performance at nearly all code lengths. Furthermore, DTCH was able to achieve convincing results even when the code length was relatively short.  Figure 3 shows a line chart plotting the average Precision@K indicator as a function of *K* for each method in performing each task. In this case, the code length was fixed at 32. It is seen that the proposed method outperformed all of the comparison methods, particularly at relatively small *K* values, and achieved significantly higher average precision values than the other methods.

## 5. Conclusion

In this paper, we proposed a supervised cross-modal hashing method called DTCH. This method simultaneously embeds a label matrix and a pairwise similarity matrix into hash learning and fully exploits the pairwise relations between samples for each label using the dual supervision approach. Specifically, to exploit the sample label matrix, the proposed method combines matrix factorization and label regression. The bidirectional mapping approach not only fully exploits the semantic information but also stabilizes the hash learning process. To exploit the pairwise similarity matrix, we adopt a semirelaxed, semidiscrete method to avoid the original nonconvex optimization problem; this also alleviates the significant cumulative quantization error that can arise from directly removing the binary constraint. We additionally designed a new out-of-sample extension strategy that is combined with the objective function's fused fine-grained features as a method for carrying out the objective function. In this manner, the consistency between the different modal distributions of samples and the pairwise similarity relations is effectively preserved. Extensive experiments carried out using two datasets verified the excellent performance and efficiency of DTCH. Furthermore, embedding deep learning in the DTCH framework as the nonlinear embedding technique slows original method. In future, we plan to investigate how to effectively and efficiently combine them.

## Figures and Tables

**Figure 1:** Framework of the proposed method.

**Figure 2:** Performance on two benchmark datasets in terms of precision score. (a) Based on MIR-Flickr. (b) Based on NUS-WIDE.

**Figure 3:** Performance on two benchmark datasets in terms of precision score with increasing *K*. (a) Based on MIR-Flickr. (b) Based on NUS-WIDE.

**Table 1:** Performance in terms of mAP score on two benchmark datasets.

Method	MIR-Flickr				NUS-WIDE			
	12 bits	16 bits	32 bits	64 bits	10 bits	16 bits	32 bits	64 bits

CVH	0.6622	0.6468	0.6771	0.6805	0.3835	0.3626	0.4055	0.4595
IMH	0.6284	0.6481	0.6395	0.6359	0.3527	0.3747	0.3801	0.3828
LSSH	0.6375	0.6511	0.6632	0.6636	0.4377	0.4313	0.4075	0.4010
SCM	0.6902	0.6958	0.7066	0.7071	0.5068	0.5545	0.4532	0.5242
DCH	0.6125	0.6238	0.5727	0.5574	0.4883	0.4989	0.5057	0.5893
FDCH	0.6711	0.6912	0.7144	0.7241	0.5195	0.5710	0.5801	0.5973
SCRATCH	**0.7315**	0.7380	0.7423	0.7560	**0.5532**	**0.5841**	**0.6197**	0.6296
TECH	0.7151	0.7215	0.7240	0.7219	0.4634	0.4552	0.5067	0.5912
Ours-1	0.7314	**0.7495**	**0.7594**	**0.7659**	0.5424	0.5424	0.6018	**0.7169**
Ours-2	**0.7497**	**0.7512**	**0.7724**	**0.8098**	**0.5836**	**0.6243**	**0.6256**	**0.7374**

CVH	0.6361	0.6409	0.6513	0.6599	0.3569	0.3591	0.3870	0.3855
IMH	0.5967	0.6131	0.6231	0.6330	0.3774	0.3903	0.4078	0.4204
LSSH	0.6619	0.6622	0.6792	0.6889	0.3980	0.4122	0.4287	0.4481
SCM	0.6947	0.7049	0.7159	0.7213	0.4978	0.5213	0.4790	0.5636
DCH	0.6465	0.6358	0.6583	0.6711	0.5266	0.5750	0.6238	0.6720
FDCH	0.7067	0.7345	0.7740	0.8006	**0.5699**	0.6123	0.6391	0.6565
SCRATCH	0.7532	0.7701	0.7805	0.7998	**0.5699**	0.5375	0.5547	0.5569
TECH	0.7399	0.7597	0.7639	0.7662	0.4608	0.4597	0.5414	0.6074
Ours-1	**0.7586**	**0.7840**	**0.7915**	**0.7999**	0.5597	**0.6697**	**0.6854**	**0.7037**
Ours-2	**0.7589**	**0.7986**	**0.8028**	**0.8249**	**0.6143**	**0.6778**	**0.6840**	**0.7593**

The upper and lower halves show the performance of Img2Text and Text2Img, respectively. Ours-1 shows the performance using DCC for optimization; Ours-2 shows the performance using DPLM for optimization. The best and suboptimal mAP values of each case are shown in boldface.

## Data Availability

The research data used to support the findings of this study are included within the article.
